RETRACTED

# AIM2 Promotes Gastric Cancer Cell Proliferation via the MAPK Signaling Pathway

**DOI:** 10.1155/2022/8756844

**Published:** 2022-04-07

**Authors:** Xiaojia Feng, Zaozhi Song, Qihui Huang, Jianguang Jia, Lingmei Zhang, Mengqi Zhu, Jun Qian

**Affiliations:** ^1^Department of Surgical Oncology, The First Affiliated Hospital of Bengbu Medical College, Bengbu, China; ^2^Department of Emergency, The Third Affiliated Hospital of Anhui Medical University, Hefei, China; ^3^Department of Oncological Gynecology, The First Affiliated Hospital of Bengbu Medical College, Bengbu, China

## Abstract

**Background:**

Gastric cancer (GC) is a highly prevalent tumor type. The dysregulated expression of melanoma deficiency factor 2 (AIM2) has been observed in a range of tumor types. Herein, we explore the role of AIM2 in the regulation of GC progression.

**Methods:**

Gastric cancer cells BGC-823 and MGC-803 in logarithmic growth phase were divided into blank group (control), Control group (NC) and SH-AIM2 group, respectively. Control group and SH-AIM2 group were transfected with AIM2 NC and SH-AIM2, respectively. Nude mice were divided into blank group (control) and SH-AIM2 group, and the treatment methods were the same as above. Differential AIM2 expression in GC tissues was assessed via bioinformatics analyses, after which western blotting was used for analyzing the AIM2 levels in tumor and paracancerous tissues from five stomach cancer patients. In addition, qPCR and protein imprinting were used to assess AIM2 expression levels in GC cells, and AIM2 knockdown was conducted in MGC-803 and BGC-823cells, after which colony formation and EdU incorporation assay were utilized to assess cell proliferation. The oncogenic role of AIM2 was then assessed in mice and validated through immunohistochemical analyses.

**Results:**

GC tissues and cell lines exhibited marked AIM2 overexpression. AIM2 knockdown significantly impaired GC cell proliferation and migration, as confirmed through *in vitro* assays. In vivo experiments showed that both the increment ability and invasion and migration ability of AIM2 knockdown group were significantly lower than that of control and NC the change of AIM2 protein level would affect the change of MAPK pathway related protein level.

**Conclusions:**

AIM2 knockdown markedly suppresses the proliferation, migration, as well as invasion of GC cells via the inhibition of MAPK signaling, thereby slowing tumor progression. Overall, these results suggest that further analyses of AIM2 may offer clinically valuable insights that can aid in the treatment of human GC.

## 1. Introduction

Gastric cancer (GC) is a substantially predominant form of cancer affecting the digestive system, and is the second common cause of death related to cancer [1]. GC incidence in China is very high, with approximately 430,000 new cases and 300,000 deaths per year [2]. The primary treatments for GC include surgical tumor removal and adjuvant radiotherapy, but 5-year survival rates remain poor in most advanced stomach cancer patients [3]. Many genes associated with the onset and progression of GC have been identified to date, but the mechanistic basis for this disease has yet to be fully defined. As such, it is vital that additional studies exploring the factors which control the development and regulation of GC be conducted in order to guide patient diagnosis and treatment.

RETRACTED

Mitogen-activated protein kinase (MAPK) family proteins are serine/threonine kinases comprising protein 38 (p38), c-Jun N-terminal kinase (JNK), and extracellular signal-regulated kinase (ERK) that are able to become activated with the aid of an extensive range of stimuli, where upon they control key cellular activities such as proliferation, mitosis, and migration [4].

Melanoma deficiency factor 2 (AIM2) is an interferon-inducible gene that is encoded on chromosome 1 in humans, and that is expressed at high levels in leukocytes in the peripheral blood, small intestine, and spleen [5] AIM2 orchestrates inflammatory responses and cell death upon parasitic infection [6, 7], but its role in oncogenic contexts remains to be clarified. There exist some facts that AIM2 can perform a dual-task in oncogenesis [8]. Early evidence from De Young et al. [5] suggested AIM2 to play a tumor suppressor role, and some researchers found that AIM2 suppressed autophagy and thereby inhibited renal cancer malignancy [9]. However, in more recent research, AIM2 was shown to be frequently mutated in colorectal neoplasms wherein It was able to inhibit neoplasia development in a manner dependent upon noninflammatory bodies [10]. AIM2 also reportedly plays a role in Epstein-Barr virus (EBV)-induced nasopharyngeal cancer development [11]. The occurrence and development of gastric cancer and various signaling pathways, gene mutations and microenvironment can regulate and participate in the process of tumor occurrence. It has been reported that AIM2 can regulate DNA-PK-Akt, MTOR-S6K1, MAPK, and other signaling pathways in colon cancer and liver cancer [10, 12, 13]. Increases in reactive oxygen species (ROS) have been detected in many cancers, and it has been reported that ROS can regulate phosphorylation activation of ERK [14], promote tumor signal transduction, and enhance cell proliferation and survival. AIM2 has been proved to induce ROS production by regulating mitochondrial dynamic balance. in addition, By regulating the dynamic balance of mitochondria, AIM2 can promote the activation of ERK by extracellular growth factor, promote the phosphorylation of Dynamin related protein 1 (DRP1), and be recruited to mitochondria to cause mitochondrial division, thus leading to the proliferation of tumor cells and drug resistance of tumor cells [15, 16] These reports further confirm that AIM2 regulates MAPK signaling pathway in no-small cell lung cancer(NSCLC)

Therefore, this paper aims to explore the interaction and relationship between AIM2 and MAPK signaling pathway in the occurrence and development of gastric cancer.

RETRACTED

## 2. Materials and Methods

### 2.1. Bioinformatics Analyses

The Cancer Genome Atlas (TCGA) database was queried for gene expression data pertaining to 375 GC patients (data type: HTseq-Counts). Genes exhibiting at least a 1-fold change in expression between GC tumor (*n* = 375) and paracancerous (*n* = 32) tissues were identified using *R*. Wilcoxon rank-sum tests were used to assess differences in AIM2 expression between these samples. Median AIM2 expression levels were used to separate patients into two groups, and ROC curves were used to assess specificity and sensitivity values associated with this cut-off value. Analyses were conducted after converting HTSEQ-FPKM data into the TPM format. Any unavailable clinical data was treated as a missing value.

### 2.2. Human Samples

All patients (*n* = 5, age 41 to 78 years, mean age about 59.5 years). In the First Affiliated Hospital of Bengbu Medical College, the patients underwent subtotal gastrectomy without preoperative radiotherapy and chemotherapy, and all patients were clearly diagnosed with primary gastric cancer. Pathological tissues and adjacent tissues were collected during operation. The study obtained the consent of the patients and was approved by the Ethics Committee of the First Affiliated Hospital of Bengbu Medical College.

### 2.3. Cell Culture and Transfection

The cell lines including MGG-803 [17], MKN-45 GC, SGC -7901, and BGC-823 [18] were provided by the Shanghai Cell Bank of the Chinese Academy of Sciences. Control GES-1 cells were from the Wuhan Pule Life Sciences Co. Ltd. (China). Culturing of all cells was carried out in DMEM (Hyclone, USA) containing penicillin/streptomycin and 10% FBS (Gibco, USA) in a 5% CO_2_ and 95% air incubator. AIM2 knockdown was achieved using shRNA constructs (AIM2: 5′-GATCCGCAAACTAT CAATCAAT CAAGAGATGTT TCAG TAGT TAGTGTTTTACGTGGTG-3′) and the pLKO .1 Lentivirus Particle Transduction system (Gene Chemistry, Shanghai, China). Cells in which AIM2 was stably knocked down were then selected for with allopurynicin, while empty lentiviral particles were used as a negative control.

RETRACTED

### 2.4. Western Blotting

Tissue samples from GC patients and controls were lysed, and total protein extracts of gastric cancer cells were analyzed by BCA method. Dilution of the samples was then carried out with 1x loading buffer, denatured at 95°C, and separated via SDS-PAGE followed by their transferring to PVDF membrane. Blots were washed thrice with TBST, blocked for 15 min with a fast block solution, and incubated overnight with primary antibodies specific for AIM2(20590-1-AP), p-ERK(ab232370), p-JNK(ab124956), ERK(ab17942), p-p38(AF4001), JNK(66210-1-Ig), and p38(66234-1-Ig) (1 : 1000; Abcam, USA) at 4°C. Blots were then washed thrice for 10 minutes per wash, succeeded by a 2 h incubation with a secondary antibody (1 : 500, Abcam, USA). After three more washes, protein bands were detected with an ECL chemiluminescence kit and scrutinized employing the Universal Gene Gel Imaging System (Syngene, Cambridge, UK).

### 2.5. qPCR

Extraction of total RNA from cells was carried out with Trizol, after which cDNA was synthesized and qPCR reactions were conducted using a standard two-step amplification program. The levels of gene expression were assessed via the 2^−ΔΔCt^ approach. Primers were synthesized by Shanghai Gene Chemicals Co. Ltd. and were as follows: AIM2-F 5′-GGCCACCATCTGTTTCTGTT-3′, AIM2-R 5′-GCCACTAAGTCAAGCTGAAATG-3′; *β*-actin-F 5′-AAGAGATGGCCACGGCTGCT-3′, *β*-actin -R 5′-TCCTTCTGCATCCTGTCGGC-3′. Thermocycler settings were as follows: 95°C, 30 s; 40 cycles of 95°C for 5 s, 60°C for 30 s. Assays were repeated in triplicate.

### 2.6. Colony Formation Assay

Cells were accumulated and replated in the plates containing 6 wells (1000 cells/well). Following incubation for 10 days, the fixation of cells with formaldehyde (4%) was carried out followed by staining with crystal violet. The colonies containing >50 cells were counted via microscope.

### 2.7. 5-Ethynyl-2-deoxyuridine (EdU) Incorporation Assay

GC cells were plated in the plates containing 24 wells until 70% confluent, at which time an EdU test kit was used based on provided directions. Briefly, cells underwent EdU labeling, fixation, Apollo staining, DAPI staining, and imaging with a fluorescent microscope, after which cells were counted using the Image-Pro software.

### 2.8. Transwell Assay

Matrigel was diluted 1 : 8 in serum-free DMEM, and 60 uL of this solution was used to evenly coat the bottom of each Transwell assay insert. Cells in the logarithmic phase of growth were then added in triplicate to inserts in serum-free media. Cells were incubated for 48 h, Cells were then counted at 200x magnification.

RETRACTED

### 2.9. Wound Healing Assays

Cells were plated in the plates containing 6 wells (5 × 105 cells/well) in triplicate until confluent, at which time a scratch wound was generated and wells were washed thrice with PBS. Cells were then cultivated for 24 h in serum-free DMEM, after which wound healing was compared between 0 and 24 h employing Photoshop. Wound Healing Rate = (1–24 h Distance/0h Range) × 100%

### 2.10. Immunohistochemistry (IHC)

Paraffin-embedded tissue sections prepared in xenograft model experiments were used for IHC analyses. probed with primary polyclonal antibodies specific for p-P38, p-JNK, or p-ERK (1 : 200, Abcam). Sections were then probed with secondary antibodies (1 : 500, Abbkine, USA) at room temperature, washed with PBS, and color development was conducted using DAB.

### 2.11. Tumor Xenografts

Male NOD-SCID mice (12 weeks old) from the Cavens Laboratory (CHangzhou, China) were randomized into control and shAIM2 groups, and were subcutaneously implanted in the flank with the corresponding GC cells (0.2 mL of a 1 × 107 cell/mL suspension in PBS). Tumor weight and diameter were measured every week for four weeks, after which mice were euthanized with 3% pentobarbital sodium, and for analysis, tumors were isolated. The Animal Experimental Ethics Committee of Bengbu Medical College approved this study.

### 2.12. Statistical Analysis

SPSS 21.0 was utilized for all statistical testing, and figures were prepared with GraphPad Prism 6.0. Outcomes are given as mean ± standard deviation (SD) while Student's *t*-tests or ANOVAs were employed for their comparison. The curves of receiver operating characteristic (ROC) were employed for assessing the diagnostic utility of AIM2 based upon area under the curve (AUC) values. *P* < 0.05 was the significance threshold, and all assessments were executed at least three times.

## 3. Results

### 3.1. GC Tissues Exhibit AIM2 Upregulation

We began by querying the TCGA database to appraise the expression of AIM2 mRNA in 375 GC tumor specimens and 32 normal gastric tissue control specimens, revealing a marked rise in AIM2 expression in tumor tissues (Figures 1(a) and 1(b)). An ROC curve revealed that AIM2 exhibited an AUC value of 52.3% (Figure 1(c)). To confirm these results, we obtained 5 pairs of GC patient tumor and paracancerous tissue from Bengbu Medical College First Affiliated Hospital. When we analyzed these samples, we confirmed that AIM2 was expressed at significantly higher levels in tumor tissues relative to matched control tissues (Figure 1(d)).

Next, Western blotting and qPCR assays were conducted which revealed marked AIM2 upregulation in SGC-7901, BGC-823, MGC803, and MKN45 in GC cells relative to control GES-1 cells (*P* < 0.05, Figures 2(a) and 2(b)). Subsequently, the expression of AIM2 in BGC823 and MGC803 cells was knocked down, as they exhibited maximal AIM2 expression in preliminary assays (*P* < 0.05, Figures 2(c) and 2(d)).

RETRACTED

### 3.2. AIM2 Promotes GC Cell Proliferation

To explore how AIM2 knockdown impacted GC cell progression, colony formation, and EdU incorporation assays were next conducted using BGC-823 and MGG-803 cells in control, NC, and sh-AIM2 treatment groups. AIM2 knockdown was found associated with an increasing reduction in colony formation (Figure 3(a)). Similarly, sh-AIM2 treatment was associated with the increasing reduction in EdU-positive cells number relative to control treatment (Figure 3(b)). Together, these data indicated that AIM2 knockdown suppresses BGC-823 and MGC 803 cell proliferation.

### 3.3. AIM2 Promotes GC Cell Invasion and Migration

Transwell and wound healing assays were next conducted to assess the relationship between AIM2 expression and GC cell migration. We found that AIM2 knockdown was associated with the decrease in the migratory activity of these cells in an assay of wound healing at 24 h (Figure 3(c)), and in the invasive activity of these wells at 48 h in a Transwell assay relative to the control and NC groups (Figure 3(d)). Overall, these findings indicated that AIM2 knockdown was sufficient to suppress GC cell invasion and migration.

### 3.4. AIM2 Knockdown Inhibits Excessive MAPK Signaling In Vitro

To explore the mechanistic basis for the above phenotypes, we next explored the effects of AIM2 knockdown on the activation of proliferation-related MAPK signaling molecules [19, 20] including P38, JNK, and ERK (Figures 4(a)–4(d)). We found that the phosphorylation of each of these three MAPKs was impaired following AIM2 knockdown in both MGC-803 and BGC823 relative to control cells.

For additional investigation of the effects of AIM2 knockdown on in vivo tumor growth, we next implanted nude mice with GC cells that had been stably transduced with lentiviral sh-AIM2 or control constructs. We observed significant decreases in tumor growth and tumor weight following AIM2 knockdown (Figures 5(a)–5(c)). We also discovered that the p-p38, p-JNK, and p-ERK levels were reduced in sh-AIM2 tumors relative to controls (Figure 5(d)), suggesting that AIM2 knockdown may inhibit excessive MAPK signaling in GC tumors, thereby constraining their growth.

## 4. Discussion

AIM2 is a cytoplasmic member of the HIN-200 family of proteins encoded on chromosome 1q22. The AIM2 protein is 344 amino acids in length and possesses an approximate molecular weight of 3,9487 Da [21] The AIM2 C-terminal domain and N-terminal domain contain HIN-200 and pyrin domains, respectively, the latter of which can bind to ASC, while the former can bind to DNA and facilitate NF-kB and Cystica1 activation, thereby inducing cell death [22]. AIM2 is involved not only in innate immune responses, but also in oncogenesis and tumor progression [8]. The AIM2 expression is highly reduced in melanoma, colorectal cancer, and prostate cancer, whereas it is upregulated in hepatocellular carcinoma, nasopharyngeal cancer, and oral squamous cell carcinoma. As such, AIM2 functions in a tumor type-specific manner [1, 8, 23, 24].

RETRACTED

Herein, we conducted bioinformatics analyses in order to evaluate AIM2 expression in GC, and we further confirmed its upregulation in GC tissues and cell lines. We therefore hypothesized that AIM2 may promote the development of GC tumors. In bioinformatics analysis, the expression of AIM2 in gastric cancer tissues was significantly increased, which was also verified in the 5 human gastric cancer tissues collected by us. Therefore, we conducted further verification in cytology and zoology. We down-regulated the expression level of AIM2 in gastric cancer cells, and found that its proliferation ability, invasion and migration ability were inhibited. In the xenotransplantation experiment, the tumor size and weight of the experimental group with down-regulated AIM2 expression level were also significantly lower than that of the blank control group. In subsequent experiments, we verified the relationship between AIM2 and MAPK signaling pathway, and the activation of MAPK signaling pathway in the group with low EXPRESSION of AIM2 was significantly inhibited. Therefore, we speculated that it was highly likely that AIM2 inhibited the activation of MAPK signaling pathway through some mechanism.

Several recent studies have clarified the role of the MAPK pathway as a key regulator of GC devlopment [25–27]. MAPK proteins are kinases that are phosphorylated in a series of steps whereupon these proteins can control key biological functions within tumor cells [28]. We found that AIM2 knockdown suppressed excessive MAPK signaling activity in GC cells, decreasing p38, JNK, and ERK phosphorylation and suppressing excessive MAPK signaling activity. However, this study also has some limitations. Our research group wants to further explore the mechanism of AIM2's influence on MAPK signaling pathway, which is similar to whether the MAPK signaling pathway is further affected by the regulation of mitochondrial dynamic balance or the production of ROS in NSCLC, which is an interesting content worth exploring.

Briefly, the findings of the current exploration show that AIM2 contributes significantly to the development and proliferation of GC cells through a mechanism dependent upon MAPK signaling, highlighting AIM2 as a viable biomarker and potential therapeutic target in GC.

RETRACTED

## Figures and Tables

**Figure 1:** AIM2 is upregulated in gastric cancer. (^*∗*^*P* < 0.05, Data obtained from three independent are represented as means and standard errors.) (a) AIM2 expression in GC tumor (*n* = 375) and paracancerous normal control tissues (*n* = 32) was assessed. (b) AIM2 expression was quantified in pairs of GC tumors and control tissues. (c) Assessment of AIM2 ROC curve sensitivity and specificity. (d) Western blotting was used to assess AIM2 protein levels in matched tumor (T) and normal (N) tissue samples. AIM2 is upregulated in GC cell lines.

**Figure 2:** Assessment and manipulation of AIM2 expression in GC cell lines (^*∗*^*P* < 0.05, Data obtained from three independent are represented as means and standard errors.) (a, b) AIM2 levels were assessed in the indicated GC cells via Western blotting and qPCR. (c, d) An shRNA construct was used to knock down AIM2 expression in GC823 and MGC 803 cells, as confirmed via qPCR.

**Figure 3:** Inhibition of GC cell malignancy by the AIM2 knockdown. (^*∗*^*P* < 0.05, Data obtained from three independent are represented as means and standard errors.) (a) BGC-823 and MGC-803 GC cells were separated into control, NC, and sh-AIM2 treatment groups and used in EdU incorporation assays to evaluate cell proliferation. (b) The average colony counts were decreased by the AIM2 knockdown in colony formation assay. (c) A wound healing assessment was employed for appraising the influences of AIM2 knockdown on GC cell migration. (d) Transwell assessments were utilized for evaluating the impact of AIM2 knockdown on GC cell invasion.

**Figure 4:** AIM2 knockdown suppresses excessive MAPK signaling activity. (^*∗*^*P* < 0.05, ^*∗∗*^*P* < 0.01, Data obtained from three independent are represented as means and standard errors.) (a-d) ERK, JNK, and P38 phosphorylation levels were assessed via Western blotting in BGC823 and MGC803 cells, with GAPDH as a normalization control. AIM2 facilitates GC tumor progression in vivo.

**Figure 5:** AIM2 knockdown suppresses *in vivo* tumor proliferation. (^*∗*^*P* < 0.05, Data obtained from three independent are represented as means and standard errors.) (a-c) Nude mice were implanted with control or AIM2-knockdown MGC803 cells. Tumor volume and weight were then measured. (d) Phosphorylated p-ERK, p-JNK and p-p38levels in control and AIM2-knockdown tumors were assessed via immunohistochemistry.

## Data Availability

The data used to support the findings of this study are available from the corresponding author upon request.

RETRACTED

## References

[1] Woerner S. M., Kloor M., Schwitalle Y. (2007). The putative tumor suppressorAIM2is frequently affected by different genetic alterations in microsatellite unstable colon cancers. *Genes, Chromosomes and Cancer*.

[2] Mendoza M. C., Er E. E., Blenis J. (2011). The Ras-ERK and PI3K-mTOR pathways: cross-talk and compensation. *Trends in Biochemical Sciences*.

[3] Zhao P., Chen D., Cheng H. (2018). Prognostic significance of soluble major histocompatibility complex class I-related chain A (sMICA) in gastric cancer. *British Journal of Biomedical Science*.

[4] Yang S.-H., Sharrocks A. D., Whitmarsh A. J. (2003). Transcriptional regulation by the MAP kinase signaling cascades. *Gene*.

[5] DeYoung K. L., Ray M. E., Su Y. A. (1997). Cloning a novel member of the human interferon-inducible gene family associated with control of tumorigenicity in a model of human melanoma. *Oncogene*.

[6] Fernandes-Alnemri T., Yu J.-W., Datta P., Wu J., Alnemri E. S. (2009). AIM2 activates the inflammasome and cell death in response to cytoplasmic DNA. *Nature*.

[7] Roberts T. L., Idris A., Dunn J. A. (2009). HIN-200 proteins regulate caspase activation in response to foreign cytoplasmic DNA. *Science*.

[8] Choubey D. (2016). Absent in melanoma 2 proteins in the development of cancer. *Cellular and Molecular Life Sciences*.

[9] Chai D., Shan H., Wang G. (2018). AIM2 is a potential therapeutic target in human renal carcinoma and suppresses its invasion and metastasis via enhancing autophagy induction. *Experimental Cell Research*.

[10] Wilson J. E., Petrucelli A. S., Chen L. (2015). Inflammasome-independent role of AIM2 in suppressing colon tumorigenesis via DNA-PK and Akt. *Nature Medicine*.

[11] Kondo Y., Nagai K., Nakahata S. (2012). Overexpression of the DNA sensor proteins, absent in melanoma 2 and interferon-inducible 16, contributes to tumorigenesis of oral squamous cell carcinoma with p53 inactivation. *Cancer Science*.

[12] Rommereim L. M., Subramanian N. (2015). AIMing 2 curtail cancer. *Cell*.

[13] Ma X., Han L. (2016). Loss of AIM2 expression promotes hepatocarcinoma progression through activation of mTOR-S6K1 pathway. *Oncotarget*.

[14] Wang G., Li Y., Yang Z., Xu W., Yang Y., Tan X. (2018). ROS mediated EGFR/MEK/ERK/HIF-1*α* Loop Regulates Glucose metabolism in pancreatic cancer. *Biochemical and Biophysical Research Communications*.

[15] Huang C.-Y., Chiang S.-F., Chen W. T.-L. (2018). HMGB1 promotes ERK-mediated mitochondrial Drp1 phosphorylation for chemoresistance through RAGE in colorectal cancer. *Cell Death & Disease*.

[16] Fu L., Dong Q., He J. (2017). SIRT4 inhibits malignancy progression of NSCLCs, through mitochondrial dynamics mediated by the ERK-Drp1 pathway. *Oncogene*.

RETRACTED

[17] Dong Z. W. (1986). [Preparation and identification of monoclonal antibody against the gastric cancer cell line MGC 803]. *Zhonghua Zhongliu Zazhi*.

[18] Deng G. R., Lu Y. Y., Chen S. M. (1987). Activated c-Ha-ras oncogene with a guanine to thymine transversion at the twelfth codon in a human stomach cancer cell line. *Cancer Research*.

[19] Li P., Xue W. J., Feng Y., Mao Q. S. (2016). Long non-coding RNA CASC2 suppresses the proliferation of gastric cancer cells by regulating the MAPK signaling pathway. *American Journal of Tourism Research*.

[20] Yang M., Huang C.-Z. (2015). Mitogen-activated protein kinase signaling pathway and invasion and metastasis of gastric cancer. *World Journal of Gastroenterology*.

[21] Asefa B., Klarmann K. D., Copeland N. G., Gilbert D. J., Jenkins N. A., Keller J. R. (2004). The interferon-inducible p200 family of proteins: a perspective on their roles in cell cycle regulation and differentiation. *Blood Cells, Molecules, and Diseases*.

[22] Man S. M., Kanneganti T.-D. (2015). Regulation of inflammasome activation. *Immunological Reviews*.

[23] Dihlmann S., Tao S., Echterdiek F. (2014). Lack of Absent in Melanoma 2 (AIM2) expression in tumor cells is closely associated with poor survival in colorectal cancer patients. *International Journal of Cancer*.

[24] Chen L. C., Wang L. J., Tsang N. M. (2012). Tumour inflammasome‐derived IL‐1*β* recruits neutrophils and improves local recurrence‐free survival in EBV‐induced nasopharyngeal carcinoma. *EMBO Molecular Medicine*.

[25] Yang G.-L., Tao H.-R., Wang H.-W. (2015). Ara-C increases gastric cancer cell invasion by upregulating CD-147-MMP-2/MMP-9 via the ERK signaling pathway. *Oncology Reports*.

[26] Akter H., Park M., Kwon O.-S., Song E. J., Park W.-S., Kang M.-J. (2015). Activation of matrix metalloproteinase-9 (MMP-9) by neurotensin promotes cell invasion and migration through ERK pathway in gastric cancer. *Tumor Biology*.

[27] Yang M., Gu Y.-y., Peng H. (2015). NAIF1 inhibits gastric cancer cells migration and invasion via the MAPK pathways. *Journal of Cancer Research and Clinical Oncology*.

[28] Yoshioka K. (2004). Scaffold proteins in mammalian MAP kinase cascades. *Journal of Biochemistry*.

